The article "College Calisthenics Teaching Based on Information Technology" was retracted in 2023. Reasons: signs of a paper mill; compromised peer review; unreliable results or conclusions.

# College Calisthenics Teaching Based on Information Technology

**DOI:** 10.1155/2022/3369743

**Published:** 2022-04-14

**Authors:** Bolong Wang

**Affiliations:** Kede College of Capital Normal University, Beijing, China

## Abstract

Under the background of national fitness, aerobics has become a popular sport. Aerobics has a good fitness effect and is one of the compulsory courses of physical education. But it also puts forward higher requirements for College Aerobics Teaching. The traditional teaching method is no longer applicable. In order to improve the teaching effect of aerobics, this paper puts forward the research of College Aerobics Teaching Method. In this paper, the traditional Aerobics Teaching Methods and the current popular information teaching mode are analyzed in detail. Through the comparison, the traditional aerobics teaching process is too boring to stimulate students' interest. But after the use of information technology teaching, students' self-learning ability has been improved. In the study of the effect of traditional teaching mode and information-based teaching mode, this paper makes relevant experimental investigation. The physical fitness of the experimental group was *P* > 0.05. There were significant differences in basic physical qualities such as push-ups, rope skipping, and flexibility between the two groups (*P* < 0.05).The experimental data show that the use of information-based teaching mode is more conducive to students' accurate grasp of action points, and because of the retrospectivity, students can consolidate knowledge and practice themselves more conveniently. The research of this paper promotes the innovation of traditional education, complements and promotes each other with traditional education, and creates greater learning and exploration space for students, in order to contribute to the construction of aerobics courses in colleges and universities.

## 1. Introduction

The state vigorously advocates quality education and is committed to promoting the all-round development of students. At the same time, put forward the slogan of national fitness; in this situation, competitive sports produced a new standard, bodybuilding operation as an important course in physical education, which should cause enough attention [1, 2]. In College Aerobics Teaching, teachers should comply with the requirements, combined with the current information technology, in order to improve the quality of teaching. As one of the advanced teaching methods, information teaching can improve the form of aerobics teaching. Therefore, it has gained more and more attention and application [3, 4].

Information-based teaching is student-centered and promotes students' autonomous learning. At the same time, it can better solve the key and difficult points in the classroom, improve learning efficiency, strengthen students' mastery of action points, and reflect the beauty of aerobics [5–7]. The information-based teaching mode has played a positive role in the aerobics curriculum in colleges and universities, effectively breaking through the limitations of the traditional classroom and opening up a new mode and road for aerobics teaching [8–10].

The article "College Calisthenics Teaching Based on Information Technology" was retracted in 2023. Reasons: signs of a paper mill; compromised peer review; unreliable results or conclusions.

This paper studies the traditional teaching methods of aerobics in colleges and universities and understands that the current traditional teaching methods of aerobics are fixed and unchanging, and the teaching methods are single, so that students' interest in learning aerobics is not high, and their enthusiasm has been hit. Therefore, this paper puts forward the research of aerobics teaching methods in colleges. In this paper, according to the characteristics of aerobics, combined with the current mainstream of information teaching methods, the traditional aerobics teaching methods are transformed and upgraded. This paper uses different teaching methods to teach aerobics to students of two classes and verifies the theory proposed by comparing the results of two classes. Through the experimental results of this paper, the data show that after using information-based teaching, the students in the experimental group have stronger learning enthusiasm, better grasp the key points of action, and the overall teaching effect is significantly improved. This paper analyzes that because of the information-based teaching to increase the richness of teaching, there is more interaction in the teaching process and through information technology to store important technical points, and students can consolidate the key points by self-study after class.

## 2. Modern Information Technology and Aerobics Teaching

### 2.1. Guiding Ideology and Task of Aerobics Teaching

#### 2.1.1. The Guiding Ideology of Aerobics Teaching

Aerobics teaching implements the new curriculum standards and new teaching guidelines, adheres to the guiding ideology of “health first, lifelong sports,” combines theory with practice, imparts knowledge, and cultivates ability. Classroom teaching and extracurricular self-study complement each other to make students healthy and innovative [11].

#### 2.1.2. Aerobics Teaching Task

1. Training students to shape beautiful posture, strong physique, and temperament
2. To develop students' physical quality, improve their coordination and sensitivity, and maintain and improve their physical and mental health [12].

Aerobics is a perfect combination of sports and art. It has the characteristics of “health, strength and beauty.” According to different learning objectives and tasks, it can be divided into three types: fitness, competitiveness, and performance. At present, aerobics has become one of the important forms of physical education, extracurricular practice, and enriching campus culture. Based on the characteristics of aerobics and its important position in sports, aerobics teaching under the background of aerobics class should fully grasp the characteristics of aerobics class and enrich the content and form of aerobics class teaching, so that learners can better master skills and cultivate aesthetic ability [13].

The article "College Calisthenics Teaching Based on Information Technology" was retracted in 2023. Reasons: signs of a paper mill; compromised peer review; unreliable results or conclusions.

### 2.2. Relationship between Modern Educational Technology and Aerobics Teaching

From the theory of teaching and education optimization, modern educational technology has a close relationship with College Aerobics Teaching. Through the theory, we can optimize the education mode and upgrade the education technology, so as to maximize the advantages of teaching effect. Creating good material conditions to ensure teaching, improving teachers' update of education methods, and optimizing education contents are the basis of improving education quality. Therefore, good teaching mode, efficient teaching tools, and means for the development of efficient aerobics have played a key role. In the field of aerobics teaching, the application of modern educational technology to assist aerobics teaching is a powerful embodiment of teaching and teaching optimization theory in teaching methods and teaching conditions [14, 15].

## 3. Experimental Objects and Methods

### 3.1. Subjects

In this experiment, a class of aerobics major in a physical education college was selected as the experimental group, and the students in class B were the control group, 8 students in each class, a total of 16 people. The experimental group used multimedia technology teaching as the main classroom teaching method, while the control group used traditional teaching as the main classroom teaching method (both groups of students were girls). The comparison results of basic physical data of the two groups are shown in Table 1.

### 3.2. Research Method

This study was made by the same aerobics' teacher according to the professional standards of aerobics course, taught the same learning content, and carried out the comparison between groups and teaching experiments. The experimental group was assisted by multimedia technology, while the control group was given priority to traditional education. The statistical analysis of relevant data verifies whether the multimedia-assisted education method is effective in classroom education. The specific experimental time and teaching arrangement are shown in Table 2.

The article "College Calisthenics Teaching Based on Information Technology" was retracted in 2023. Reasons: signs of a paper mill; compromised peer review; unreliable results or conclusions.

## 4. Discussion

### 4.1. Experimental Results and Analysis

It can be seen from Figures 1 and 2 that before the experiment, the physical fitness of the two groups was *P* > 0.05. There were significant differences between the two groups in terms of basic physical fitness such as push-up, rope skipping, and flexibility (*P* < 0.05), indicating that information-based teaching is more suitable for aerobics teaching than traditional teaching. This is because multimedia can also be used to assist after-school teaching, so that teachers can supervise students to complete the exercises after class, so that students can practice more actively after class.

After the experiment, the data of the experimental group and photos were counted, as shown in Figures 3 and Figures 4. From the statistical results, it can be seen that in addition to the static impact on the right angle support, the three groups of movements are jumping, balance, and flexibility difficulty movements, and the final score of the two groups is *P* < 0.05. It shows that multimedia-assisted teaching technology has more advantages in the teaching process of dynamic and difficult movements.

### 4.2. Analysis of the Concept of Information Teaching and Traditional Teaching Mode

#### 4.2.1. The Concept of Information Teaching

Information-based education refers to the technology based on the Internet, which can be applied to practical teaching and achieve good learning effect. Especially under the education department's attention, information teaching has become an indispensable part of education. For example, microlecture, QQ, WeChat discussion group, and video have become very important information sources in teaching. Information teaching provides more knowledge sources for students and greatly improves learning efficiency.

#### 4.2.2. Traditional Education Mode

The traditional education mode can be divided into preparation part, basic part, and ending part. Teaching is generally in accordance with these three parts to complete; the basic steps of each class are the same; education methods are relatively simple, over time, greatly reducing students' interest in learning.

### 4.3. Characteristics of Information Technology and Application of Aerobics Teaching

Aerobics education based on modern information technology has achieved good results. Through the use of technology in classroom education, relevant theoretical knowledge and important operations can be more intuitive, vivid, and vivid in front of students. Teachers can explain the key knowledge in detail, and video equipment can record the whole teaching process, providing convenience for teachers and students. Microsystem provides a more powerful analysis and feedback tool for teachers and students, and the advantages of modern technology itself will be better displayed.

The article "College Calisthenics Teaching Based on Information Technology" was retracted in 2023. Reasons: signs of a paper mill; compromised peer review; unreliable results or conclusions.

### 4.4. Using “Information” Teaching to Achieve Teaching Objectives Effectively

In information teaching, teachers can change their teaching methods and use network information teaching equipment and rich music resources to stimulate students' enthusiasm for sports. Rich video resources and fashionable and happy body language let students involuntarily into the classroom.

#### 4.4.1. Improve the Enthusiasm of Students to Participate in Sports

Before aerobics education, teachers should guide students to watch the aerobics performance video on the electronic screen. The performers are energetic, elegant, fluent, and rhythmic. Under such visual impact, students will unconsciously be interested in aerobics, so as to actively participate in the study and practice of aerobics and lay the foundation for lifelong love of aerobics.

#### 4.4.2. Provides the Possibility to Watch and Practice Repeatedly

Teachers can use information education equipment in teaching, upload the learning content to the network before class, and students can watch and practice in their spare time, so as to realize the “image action” in the heart. In class, teachers can show the content they need to teach in the form of video, so that students know the route of each movement and the movements of each part of the body. After finishing a group of movements, students should coordinate their head, neck, shoulder, upper limbs, and chest and improve their flexibility, coordination, bouncing, balance, and other physical qualities. Through repeated watching and practice, students can effectively master the movement skills and effectively complete the teaching objectives.

#### 4.4.3. Group Teaching after Class Is Conducive to Self-Study

Team work, independent inquiry, innovative consciousness, and independent problem-solving ability are the necessary abilities for students to enter the society. In teaching, teachers can organize students into groups, and the team members can make use of information teaching resources such as decomposition action video to carry out independent inquiry learning.

### 4.5. Fashion of Teaching Content Selection

The content of aerobics practice course should not only be rich, but also be connected with fashion. To improve their interest and update the education content is the core of education reform. Aerobics itself is inclusive and presents in front of people in a variety of styles and postures, giving dynamic and expressive action. In the new era, college students pursue fashion and new concepts. Therefore, fashion content should be added to the basic content, such as the latest warm-up action in the preparation part. In the basic technology part, in addition to teaching a complete set of aerobics, we can also add dance contents such as Latin dance.

The article "College Calisthenics Teaching Based on Information Technology" was retracted in 2023. Reasons: signs of a paper mill; compromised peer review; unreliable results or conclusions.

## 5. Conclusions

With the vigorous development of “Internet plus education,” the integration of educational resources and the continuous optimization of teaching platforms will greatly enrich the content and form of aerobics information teaching. At that time, aerobics teaching can make systematic personalized courses by using VR and other high-tech tools according to different audiences, so as to meet the learning demands of different audiences. Through the experimental data, it can be seen that the control group using traditional education is obviously weaker than the experimental group using information-based teaching. This paper analyzes that information-based education can effectively improve the effect of aerobics education, and it is easier to achieve the goal of aerobics teaching. Information technology is an education method, but based on this technology, the expansibility of aerobics teaching has been greatly improved, which is more in line with the current is education requirements than the traditional teaching mode.

## Figures and Tables

**Figure 1:** Physical fitness statistics of experimental group.

**Figure 2:** Physical fitness statistics of the control group.

**Figure 3:** Statistics of difficulty movement test results of experimental group after experiment.

**Figure 4:** Statistics of difficulty movement test results in control group after experiment.

**Table 1:** Basic information of experimental group and control group.

Group	Number of people	Age/age	Height/cm	Weight/kg
Experience group	8	19.67 ± 0.38	163.17 ± 1.18	51.74 ± 0.57
Control group	8	19.89 ± 0.41	162.79 ± 1.15	51.19 ± 0.52

**Table 2:** Experiment time and teaching arrangement.

Teaching time	Teaching week	Class hour	Teaching time
March-June 2019	4 weeks per month for a total of 16 weeks	Three times a week, two hours a time, a total of 96 hours	Each teaching time is 100 minutes

## Data Availability

The data underlying the results presented in the study are available within the manuscript.
